# Human endometrial cell coculture reduces the endocrine disruptor toxicity on mouse embryo development

**DOI:** 10.1186/1745-6673-7-7

**Published:** 2012-04-30

**Authors:** Myeong-Seop Lee, Young-Sang Lee, Hae-Hyeog Lee, Ho-Yeon Song

**Affiliations:** 1 Department of Microbiology, School of Medicine, Soonchunhyang University, Cheonan, 330-090, South Korea; 2 Industry Academy Cooperation Foundation, Soonchunhyang University, Asan, 336-745, South Korea; 3 Department of Biomedical Technolgy, Soonchunhyang University, Asan, 336-745, South Korea; 4 Department of Obstetrics and Gynecology, Soonchunhyang University Bucheon Hospital, Bucheon, 420-767, South Korea

**Keywords:** Bisphenol A, Aroclor 1254, Mouse embryo, Human endometrial cells, Endocrine disruptors

## Abstract

**Backgrounds:**

Previous studies suggested that endocrine disruptors (ED) are toxic on preimplantation embryos and inhibit development of embryos *in vitro* culture. However, information about the toxicity of endocrine disruptors on preimplantation development of embryo in human reproductive environment is lacking.

**Methods:**

Bisphenol A (BPA) and Aroclor 1254 (polychlorinated biphenyls) were used as endocrine disruptors in this study. Mouse 2-cell embryos were cultured in medium alone or vehicle or co-cultured with human endometrial epithelial layers in increasing ED concentrations.

**Results:**

At 72 hours the percentage of normal blastocyst were decreased by ED in a dose-dependent manner while the co-culture system significantly enhanced the rate and reduced the toxicity of endocrine disruptors on the embryonic development *in vitro*.

**Conclusions:**

In conclusion, although EDs have the toxic effect on embryo development, the co-culture with human endometrial cell reduced the preimplantation embryo from it thereby making human reproductive environment protective to preimplantation embryo from the toxicity of endocrine disruptors.

## Backgrounds

Endocrine disruptors are man made chemicals that have been shown to affect reproduction in wild life and may have adverse effects on humans [1-3]. Bisphenol A (BPA) is an important monomer used in the manufacture of a large number of chemicals and products, including epoxy and polystyrene resins that are used frequently in the food-packaging industry and in dentistry. Polychlorinated biphenyls (PCBs), a family of 209 highly stable synthetic congeners, were used for a decade in a wide range of industrial applications, due to their excellent flame retardant, lubricant, and electrical insulating properties.

Human exposure to these chemicals is significant. BPA have been detected in liquid from canned vegetables [4] and in the saliva of patients treated with dental sealants [5]. The wide spread use and high chemical stability make PCBs ubiquitous and persistent in nature and their high lipophilicity causes these compounds to bio-accumulate, with the food chain being the main route of exposure. Especially, embryos, fetuses and newborns are highly susceptible to the exposure of these chemicals, which highlights the developmental toxicity of the compounds [6,7]. Further examples of exposure of human endometrium to the endocrine disruptors was demonstrated elsewhere although the levels were negligible [8]. Individual congener and total PCB concentrations were determined in serum (819–2627 pg/g whole weight) and follicular fluid (303–1257 pg/g whole weight) obtained from women undergoing assisted reproductive technologies (in vitro fertilization and embryo replacement) [9].

Endometrium is the main target for estrogens besides the breast, the pituitary, and the hypothalamus, and thus endometrium could be a useful tissue for evaluating the relevance of environmental estrogen exposure. Endometrial tissue is vital to important biological processes such as implantation and embryonic to blastocyst development, and disturbances in the function of this organ can lead to reduced fertility [8].

Embryos might be more sensitive to the endocrine disruptors than fetuses because preimplantation exposure might cause direct contact of endocrine disruptors that had entered maternal tissues, without placental barriers [10]. However, there remains a lack of knowledges about development of preimplantation embryos at the earliest stages in the presence of endocrine disruptors on human endometrium. So far, monolayers of purified epithelial cells or polarized epithelial cells have been used to investigate the effects of various materials on embryo development [11,12]. In a recent study, it was found that BPA partly affects implantation sites and alter the expression of implantation-associated genes [13]. Berger RG et. al. also showed that BPA exposure disrupts intrauterine implantation during early gestation [14]. However, the effects of BPA or BCP on the development of mouse embryos in presence or absence of human endrometrium epithelial cell have not been evaluated which can be interesting to understand the protective effect of embryos in cohort of co-culture system in vivo. In this study, we investigated the effects of two known endocrine disruptors, BPA or Aroclor 1254 (a commercial PCB; contains biphenyls with approximately 54% chlorine) on the development of mouse embryos (2-cells) co-cultured on human endometrial epithelial cell (hEEC) monolayers as an *in vivo* model by examination of dose dependency on embryo development.

## Methods

### Human endometrial epithelial (hEEC) cell culture

To study the development of mouse embryos under toxic exposure and their protective measures in vitro, toxic endocrine disruptors such as BPA or Arocolor-1245 were used on mouse embryos. Therefore, this study was first approved by the Institutional Review Board (IRB) of Soonchunhyang University Hospital, South Korea (IRB no. SCH 2009–36).

Human endometrial tissues were collected from normal cycling patients of the proliferative stages (days 4–14) who had undergone hysterectomy for uterine myoma at the Department of Obstetrics and Gynecology, Soonchunhyang University Hospital, from April 1 to July 30, 2009. For isolation and primary culture of human endometrial epithelial cells (hEECs), endometrial samples were processed following the method described by Ryan *et al*. [15] with minor modifications. Briefly, minced endometrial tissue was digested with collagenase (2 mg/ml; Gibco BRL, Grand Island, NY) at 37°C in Ca^++^, Mg^++^-free PBS (Gibco, Carlsbud, CA, USA) for about 1 hr. Further mechanical separation was performed by repeated suction by pipetting. The suspension was serially filtered through a 100-μm cell strainer (Falcon, Franklin Lakes, NJ, USA) and a 40-μm cell strainer (Falcon). hEECs were backwashed from the 40-μm cell strainer with the PBS and freed of collagenase by centrifugation (600 g, 5 min). The cell pellet was resuspended in phenol red-free M199 (Gibco) containing antibiotics that was supplemented with 10% charcoal-dextran-treated fetal bovine serum (Hyclone Laboratories, South Logan, UT), 1nM E_2_ (Sigma-Aldrich, St. Louis, MO, USA) and Insulin-Transferrin Sodium selenite (5 μg/ml; Sigma-Aldrich). This medium was also used for embryo culture. Cell density was determined in a Neubauer hemocytometer. The cells were seeded on 4-well dishes and cultured until confluency at 37^0^ C in a humidified atmosphere of 5% CO_2_ in air. The epithelial cells later grew as whorl around the explants (Figure 1) and cell viability was greater than 90%. After reaching 80% confluence in medium cells were found polyhedral in shape and epithelioid characteristics of epithelial cells. The homogeneity of cultures was determined by morphologic characteristics and verified by immunocytochemical localization of cytokeratin, vimentin, as described elsewhere [16]. After primary culture (day 4) cells were examined. Antiserum to cytokeratin reacted strongly with EEC and revealed the characteristic cytoarchitecture showing intermediate filamentous orientation of cytokeratins. 

**Figure 1:** Morphology of human endometrial epithelial cells isolated freshly (a), attached (b) and confluent (c) (X100).

### Retrieval of mouse 2-cell embryos and Endocrine disruptor treatments

A total of 149 mice were used in this study, 75 of which for PCB and 74 for BCP. Five-week-old ICR female mice (from Korea Research Institute of Bioscience and Biotechnology, Daejeon, Korea) were injected with 10 IU of intraperitoneal pregnant mare serum gonadotropin and with 10 IU intraperitoneal human chorionic gonadotrophin (hCG) 48 hrs later. They were impregnated overnight by 12-week-old males of the same strain. Mating was ascertained by the appearance of a vaginal plug on the following morning. Female mice were killed at 48 hr after hCG administration by cervical dislocation and mouse 2-cell embryos were flushed from the oviducts.

Mouse 2-cell embryos were cultured in the medium for 72 hrs in increasing BPA (Sigma-Aldrich) concentrations (0, 10^−8^, 10^−6^, 10^−4^ M) or Aroclor 1254 (200 μg/ml dissolved in methanol; Supelco) concentrations (0, 0.02, 0.2, 1 μg/ml) to investigate the dose dependent toxicities of BPA and Aroclor 1254 on the embryonic development. The concentration of 0 M (BPA) or 0 μg/ml (Aroclor 1254) was control group. The percentages of blastocyst were determined as the rate of development of blastocyst at 72 hour (Figures 2, 3). The E_2_ and BPA were dissolved in ethanol as stock solutions and Aroclor 1254 in methanol. The concentration of vehicle solution added into the culture medium was 0.01% (ethanol) or 0.05% (methanol), respectively. Co-culture was done with the hEEC monolayer in the medium as described above. Blastocysts were stained with Hoechst 33342 and the number of cells in the blastocysts was counted to determine whether degenerated or not (Figure 4).

**Figure 2:** Morphology of mouse embryos developed normally in the medium (a) or the coculture (b) (X100).

**Figure 3:** Morphology of mouse embryos degenerated by endocrine disruptors in the medium (a) or the coculture (b) (X100).

**Figure 4:** Fluorescence micrograph of normal (a) and abnormal (b) mouse blastocyst stained with Hoechst 33342 (X400).

### Statistical analysis

Ki square test was performed on the data in order to determine significant differences (P < 0.05) between the treatment (media contains a series of increasing concentrations of endocrine disruptors) and control (not treated with any of the endocrine disruptors; i.e. - media contains null/zero concentration of endocrine disruptors) groups.

## Results

To investigate the toxicological impact of endocrine disruptors (BPA or Aroclor 1254) and the effect of human reproductive environment, dose dependent concentrations of the endocrine disruptors were exposed on mouse 2-cell embryos cultured in the medium or on hEEC monolayers and the embryonic development was compared to that of control (media without any endocrine disruptors). Tables 1 and 2 showed the dose dependent toxicities of BPA and Aroclor 1254 on the preimplantation development of embryos and the protective effect of human reproductive environment on preimplantation embryos.

**Table 1:** The effect of coculture on development of mouse embryos in increasing Bisphenol A

**Concentrations** ** (M)**	Embryos grown on*	**Total number of embryos**	**Number of blastocysts**	**% of** **blastocyst**^**a**^
0	Medium alone	125	116	93
	Vehicle	144	130	90
	Coculture	112	110	98^b^
10^−8^	Medium alone	121	102	84
	Vehicle	132	107	81
	Coculture	123	111	90^b^
10^−6^	Medium alone	120	80	67
	Vehicle	123	76	62
	Coculture	121	87	72^b^
10^−4^	Medium alone	135	0	0^c^
	Vehicle	113	0	0^c^
	Coculture	123	62	50^bc^

*Mouse embryos were grown on three different kinds of culture system. In Medium alone M199 (Gibco) media were used. In Vehicle, vehicle solutions (ethanol/methanol) were used. In co-culture, embryos were grown on human endometrial epithelial cells (hEECs).

^a^The percentages of blastocyst at 72hour of culture.

^b^Values in coculture were significantly higher than those in medium alone, respectively: *P* < 0.05.

^c^Values were significantly lower than those of each control(0 μg/ml), respectively: *P* < 0.05.

**Table 2:** The effect of coculture on development of mouse embryos in increasing Aroclor 1254 concentrations

**Concentrations** ** (μg/ml)fs**	**Group**	**Total number of embryos**	**Number of blastocysts**	**% of** **blastocyst**^**a**^
0	Medium alone	122	111	91
	Vehicle	113	102	90
	Coculture	133	125	94^b^
0.02	Medium alone	133	109	82
	Vehicle	121	97	80
	Coculture	125	110	88^b^
0.2	Medium alone	121	76	63
	Vehicle	115	69	60
	Coculture	120	82	68^b^
1	Medium alone	122	0	0^c^
	Vehicle	119	0	0^c^
	Coculture	128	55	43^bc^

*Mouse embryos were grown on three different kinds of culture system. In Medium alone M199 (Gibco) media were used. In Vehicle, vehicle solutions (ethanol/methanol) were used. In co-culture, embryos were grown on human endometrial epithelial cells (hEECs).

^a^The percentages of blastocyst at 72hour of culture.

^b^Values in coculture were significantly higher than those in medium alone, respectively: *P* < 0.05.

^c^Values were significantly lower than those of each control(0 μg/ml), respectively: *P* < 0.05.

### Effect of BPA

From Table 1 it was clear that BPA at 10^−4^ M concentrations had the greatest detrimental effect on the development of embryos at 72 hour of culture. No blastocyst was observed in case of both medium alone and vehicle and only 50% blastocysts were observed for coculture system (p < 0.05). It was also evident that when the concentration of BPA was increased, the total number of blastocysts was also decreased. However, coculture with hEEC monolayers was found to be beneficial because the decreasing rate of blastocysts number was much smaller than that of the medium or vehicle (Table 1).

### Effect of Aroclor 1254

Similar dose dependent effect of Aroclor 1254 at different concentrations was observed on embryonic development in Table 2. The detrimental effect of Aroclor 1254 on embryonic development was found to be increasing with the increase of concentration in all treatment groups at 72 hour. Especially, 1 μg/ml Aroclor 1254 showed the most detrimental effect. In this concentration only 43% blastocysts were observed for co-culture system, but none for media alone and vehicle (P < 0.05). Also in this case, co-culture was found beneficial by decreasing the rate of detrimental effect Aroclor 1254 on embryonic development (Table 2). Thus these results showed that the hEEC coculture alleviated the toxicity of BPA or Aroclor 1254 on the embryonic development, especially in the high dose.

## Discussion

Three different types of cells, e.g. – the epithelium, the endometrial stroma and the myometrium, are known to found in mammalian uterus. The differentiation of endometrial epithelia is considered important regarding successful embryonic development, placentation or embryo implantation. But due to environmental pollution and extensive distribution of PCBs in the ecosystem, endometrial cells have over exposed to these carcinogenic chemicals and several studies have reported the detrimental effects PCBs on animal reproduction systems. In human beings, complications such as reduced birth weight, diminished head circumference and reduced gestational age have been reported to occur due to maternal consumption of PCB contaminated fish [17,18]. Among various chemical formulations, BPA and Aroclor 1254 are the known endocrine disruptors of the PCB family.

To date, several studies have indicated that BPA mimics estrogen and 10^−8^ to 10^−6^ M BPA exerts estrogenic effects on various kind of cells in vitro [10,14,19] and over 10^−5^ M BPA is cytotoxic [20]. On the other hand, one to 10 μg/ml Aroclor 1254 was found cytotoxic [21-23].

In this study, endocrine disruptors decreased the developmental rates of embryos by dose dependency (Table 1, 2). Takai *et al*[10]. have shown that BPA significantly decreased the developmental rate of two-cell mouse embryos to blastocysts in vitro. Kholkute *et al*. [21,22] examined the effect of Aroclor 1254 on the development of 2-cell embryos to the 4-cell stage at 48 hr. They found that increasing the concentration of Aroclor 1254 in the culture medium significantly reduced the progression of 2-cell embryos to the 4-cell stage or greater at 48 hr. Also, the presence of Aroclor 1254 reduced both the in vitro fertilization rates and embryonic development in mice. The results demonstrated that increasing concentrations of BPA or Aroclor 1254 had a deleterious effect directly on embryonic development.

During the blastulation, differentiation events were occurred and contact-induced cell polarization and reorganization of cytoskeletal elements were expressed. In this study, the blastulation at 72 hr in the medium alone and vehicle was not observed at 10^−4^ M (BPA) or 1 μg/ml (Aroclor 1254). It might be due to the fact that the chemicals have aneuploidogenic properties that inhibit MT assembly in intact cells. Pfeiffer *et al*. [24] demonstrated by staining with anti-centromere antibodies that all micronuclei in V79 cells induced by BPA contained whole chromatids/chromosomes, suggesting that BPA does not induce DNA breakage. Tsutsui *et al*. [25] reported that BPA exerted transforming and genotoxic effects on cultured syrian hamster embryo (SHE) cells and the DNA adduct formation observed in cultured SHE cells treated with BPA was involved in non-disjunction, leading to aneuploidy. Takai *et al*. [26] demonstrated that embryos that did not reach the blastocyst stage at 48 hrs were largely in the morula stage, although the percentage of degenerated embryos was significantly increased in the 10^−4^ M BPA-exposed group. Hernandez and Dukelow reported that the morula was more susceptible to the toxic effect of Aroclor 1254 and Aroclor 1254 could affect the development of the embryos by reducing the number of gap junctions [23]. Several other studies indicate that even human endometrial cells are susceptible to the exposure of ED [27,28]. In this study, BPL and Aroclor 1254 might have some toxic effect on hEEC too, but co-culturing mouse embryos with hEEC monolayer cells is advantageous.

The beneficial effects of co-culture include the secretion of embryotrophic factors such as nutrients and substrates, growth factors and cytokines and the removal of potentially harmful substances such as heavy metals, ammonium, and free radical formation, detoxifying the culture medium [29]. In this study, the co-culture with hEECs increased the percentages of blastocyst in all treatments. However, it should be noted that the total cell in co-culture system might be higher than that of the medium alone or vehicle. Therefore, decreasing the BPA or Arocolor-1245 concentration in the co-culture system might have a reduced toxic effect as compared with medium alone or vehicle culturing. In other cases, bio-transformation of these chemicals causes bio-accumulation in increased concentrations.

Because of ethical and legal issues, an in vitro model was used to elucidate the impacts of endocrine disruptors on embryonic development. The results should be considered in light of the limitations of an in vitro model. In addition, mouse embryos were used rather than human embryos. Nevertheless, the results from this study were useful in evaluating impacts of endocrine disruptors at the human endometrial-embryonic interface.

## Conclusions

In conclusion, increasing concentrations of BPA or Aroclor 1254 had a deleterious effect directly on embryonic development. This suggests that the endocrine disruptors, BPA and Aroclor 1254 might dose dependently reduce the embryo development on reproductive environment. However, in this study, we showed mouse endometrial cell coculture reduced the toxicities of BPA and Aroclor 1254 on preimplantation development of embryos and this suggests that reproductive environment protects preimplantation embryo from the toxicity of endocrine disruptor.

## Competing interests

The authors report no competing interests with any person or institution.

## Authors’ contributions

M-S L and H-Y S provided the idea for the study. M-S L, Y-S L, H-H L did in vitro works; M-S L, Y-S L, H-H L and Y-S L analyzed and interpreted the data. M-S L and H-Y S wrote the paper. All authors revised it and approved the version to be published. H-Y S is the guarantor. All authors read and approved the final manuscript.

## References

[B1] ColbornTvom SaalFSSotoAMDevelopmental effects of endocrine-disrupting chemicals in wildlife and humansEnviron Health Perspect199310137838410.1289/ehp.931013788080506PMC1519860

[B2] DastonGPEnvironmental estrogen and reproductive health: a discussion of the human and environmental dataReprod Toxicol19971146548110.1016/S0890-6238(97)00014-29241667

[B3] SonnenscheinCSotoAMAn updated review of environmental estrogen and androgen mimics and antagonistsJ Steroid Biochem Mol Biol19986514315010.1016/S0960-0760(98)00027-29699867

[B4] BrotonsJAXenoestrogens released from lacquer coatings in food cansEnviron Health Perspect199510360861210.1289/ehp.951036087556016PMC1519121

[B5] OleaNEstrogenicity of resin-base composites and sealants used in dentistryEnviron Health Perspect199610429830510.1289/ehp.961042988919768PMC1469315

[B6] KimJCEvaluation of developmental toxicity in rats exposed to the environmental estrogen bisphenol A during pregnancyLife Sci2001692611262510.1016/S0024-3205(01)01341-811712665

[B7] ColettiDPolychlorobiphenys inhibit skeletal muscle differentiation in cultureToxicol Appl Pharmacol200117522623310.1006/taap.2001.923711559021

[B8] SchaeferWRExposure of human endometrium to environmental estrogens, antiandrogens, and organochlorine compoundsFertil Steril20007455856310.1016/S0015-0282(00)00704-410973655

[B9] PauwelsAThe relation between levels of selected PCB congeners in human serum and follicular fluidChemosphere1999392433244110.1016/S0045-6535(99)00170-810581696

[B10] TakaiYEstrogen receptor-mediated effects of a xenoestrogen, bisphenol A, on preimplantation mouse embryosBiochem Biophys Res Commun200027091892110.1006/bbrc.2000.254810772925

[B11] CarrascoICebralEBenitezRVantmanDHydrosalpinx fluid affects murine embryonic development in a coculture system with epithelial endometrial cellsFertil Steril2001751004100810.1016/S0015-0282(01)01683-111334916

[B12] ValbuenaDIncreasing levels of estradiol are deterious to embryonic implantation because they directly affect the embryoFertil Steril20017696296810.1016/S0015-0282(01)02018-011704118

[B13] VarayoudJRamosJGBosquiazzoVLLowerMMunoz-de-ToroMLuqueEHNeonatal exposure to bisphenol A alters rat uterine implantation-associated gene expression and reduces the number of implantation sitesEndocrinology201115231101111110.1210/en.2009-103721285323

[B14] BergerRGFosterWGde CatanzaroDBisphenol-A exposure during the period of blastocyst implantation alters uterine morphology and perturbs measures of estrogen and progesterone receptor expression in miceReprod Toxicol201030339340010.1016/j.reprotox.2010.06.00620599497

[B15] RyanIPSchriockEDTaylorRNIsolation, characterization, and comparison of human endometrial and endometriosis cells in vitroJ Clin Endocrinol Metab19947864264910.1210/jc.78.3.6428126136

[B16] PierroEStromal-epithelial interactions modulate estrogen responsiveness in normal human endometriumBiol Reprod20016483183810.1095/biolreprod64.3.83111207198

[B17] FeinGGPrenatal exposure to polychlorinated biphenyls: effects on birth size and gestational ageJ Pediatr198410531532010.1016/S0022-3476(84)80139-06431068

[B18] SwainWREffects of organochlorine chemicals on the reproductive outcome of humans who consumed contaminated great lake fish: an epidemiological considerationJ Toxicol Environ Health19913358763910.1080/152873991095315411908527

[B19] KrishnanABisphenol-A: an estrogenic substance is released from polycarbonate flasks during autoclavingEndocrinology19931322279228610.1210/en.132.6.22798504731

[B20] NakagawaYTayamaSMetabolism and cytotoxicity of bisphenol A and other bisphenols in isolated rat hepatocytesArch Toxicol2000749910510.1007/s00204005065910839477

[B21] KholkuteSDRodriguezJDukelowWRReproductive toxicology of Aroclor-1254: effects on oocyte, spermatozoa, in vitro fertilization, and embryo development in the mouseReprod Toxicol1994848749310.1016/0890-6238(94)90031-07881200

[B22] KholkuteSDRodriguezJDukelowWREffects of polychlorinated biphenyls (PCBs) on in vitro fertilization in the mouseReprod Toxicol19948697310.1016/0890-6238(94)90069-88186627

[B23] HernandezODukelowWRAroclor-1254 effects on the in vitro development of 8-cell mouse embryosBul Environ Contam Toxicol19986077378010.1007/s0012899006939595194

[B24] PfeifferERosenbergBDeuschelSMetzlerMInterference with microtubules and induction of micronuclei in vitro by various bisphenolsMut Res1997390213110.1016/S0165-1218(96)00161-99150749

[B25] TsutuiTBisphenol-A induces cellular transformation, aneuploidy and DNA adduct formation in cultured Syrian hamster embryo cellsInt J Cancer19987529029410.1002/(SICI)1097-0215(19980119)75:2<290::AID-IJC19>3.0.CO;2-H9462721

[B26] TakaiYPreimplantation exposure to bisphenol A advances postnatal developmentReprod Toxicol20011571741113738010.1016/s0890-6238(00)00119-2

[B27] AghajanovaLGiudiceLCEffect of bisphenol A on human endometrial stromal fibroblasts in vitroReprod Biomed Online201122324956Epub 2010 Dec 2310.1016/j.rbmo.2010.12.00721273127PMC3836676

[B28] BredhultCBacklinBMOlovsson M Effects of some endocrine disruptors on the proliferation and viability of human endometrial endothelial cells in vitroReprod Toxicol200723455055910.1016/j.reprotox.2007.03.00617493787

[B29] BavisterBDCulture of preimplantation embryos: facts and artifactsHum Reprod Update199519114810.1093/humupd/1.2.9115726768

